The article "RBFOX3 Promotes Gastric Cancer Growth and Progression by Activating HTERT Signaling" was retracted in 2021. Reason: concerns about the images.

# RBFOX3 Promotes Gastric Cancer Growth and Progression by Activating HTERT Signaling

**DOI:** 10.3389/fonc.2020.01044

**Published:** 2020-07-20

**Authors:** Chen Luo, Xiaojian Zhu, Qilin Luo, Fanqin Bu, Chao Huang, Jingfeng Zhu, Jiefeng Zhao, Wenjun Zhang, Kang Lin, Cegui Hu, Zeng Zong, Hongliang Luo, Jun Huang, Zhengming Zhu

**Affiliations:** ^1^Department of General Surgery, The Second Affiliated Hospital of Nanchang University, Nanchang, China; ^2^Department of Clinical Medical, Jiangxi Medical College of Nanchang University, Nanchang, China; ^3^Jiangxi Province Key Laboratory of Molecular Medicine, Nanchang, China

**Keywords:** RBFOX3, HTERT, gastric cancer, promoter-binding protein, cancer biomarker

## Abstract

Tumor invasion, metastasis, and recrudescence remain a considerable challenge in the treatment of gastric cancer (GC). Herein we first identified that RNA binding protein fox-1 homolog 3 (RBFOX3) was markedly overexpressed in GC tissues and negatively linked to the survival rate of GC patients. RBFOX3 promoted cell division and cell cycle progression *in vitro* and *in vivo*. Furthermore, RBFOX3 increased the cell invasion and migration ability. The suppression of GC cell multiplication and invasion, caused by silencing of RBFOX3, was rescued by HTERT overexpression. Additionally, RBFOX3 augmented the resistance of GC cells to 5-fluorouracil by repressing RBFOX3. Mechanistically, the exogenous up-regulation of RBFOX3 triggered promoter activity and HTERT expression, thereby enhancing the division and the development of GC cells. Further co-immunoprecipitation tests revealed that RBFOX3 bound to AP-2β to modulate HTERT expression. In conclusion, our study indicates that a high expression of RBFOX3 promotes GC progression and development and predicts worse prognosis. Collectively, these results indicate that the RBFOX3/AP-2β/HTERT signaling pathway can be therapeutically targeted to prevent and treat GC recurrence and metastasis.

## Introduction

Gastric cancer (GC) is the third leading cause of cancer deaths worldwide and the most common gastrointestinal malignancy in East Asia and Latin America (1). China has seen a rise in the cases of GC, which has been attributed to lifestyle and dietary changes (2). Despite that the diagnosis and the treatment of GC have made remarkable progress, GC prognosis remains poor, with a low 5-year survival rate, due to disease recurrence and high metastasis rate (3). The pathogenesis of GC is highly complex and poorly understood. Genetic factors, *Helicobacter pylori* infection, unhealthy eating habits, and smoking are all involved in the development of GC (4). Owing to the complexity of the abdominal microenvironment, GC recurrence is relatively high, and further treatment does not effectively improve the patients' quality of life. Thus, investigating the molecular mechanisms of GC tumorigenesis and progression is imperative to develop more effective prevention and treatment options.

RNA binding protein fox-1 homolog 3 (RBFOX3) is a member of Fox1 family which can be encoded by the *Rbfox3* gene on chromosome 17 and encodes 15 exons (5). In mammals, this family of splicing factors consists of three members. RBFOX1 is abnormally increased in the heart, neural tissues, and skeletal muscles. RBFOX2 exhibits a broader expression pattern, occurring in embryos, neurons, and muscles. However, RBFOX3 is expressed in neurons under physiological conditions (6, 7). RBFOX3 regulates brain-specific pre-mRNA splicing choices by binding to RNA penta/hexa nucleotide UGCAUG motif (8). Furthermore, it also interacts with the polypyrimidine tract-binding protein-associated splicing factor (PSF) (9), which increases the RBFOX3 binding target UGCAUG motif (10). However, recent studies suggest that RBFOX3 modulates various pathological processes. Evidence suggested that neuronal nuclei (NeuN) is a product of RBFOX3, which can serve as a marker in post-mitotic neurons (11). Moreover, previous studies have shown that RBFOX3 could bind to DNA (12, 13). RBFOX3 has also been reported to control the biogenesis of some miRNAs, such as primary-miRNAs (pri-miRNAs), that lack a UGCAUG motif (14). We hypothesized that, in addition to its splicing functions, RBFOX3 regulates various biochemical processes that are poorly understood. Here we find that RBFOX3 promotes GC by regulating HTERT expression. We find that RBFOX3 is significantly up-regulated in GC and that it correlates with poor survival. Functional analyses revealed that RBFOX3 enhances GC growth, metastasis, and chemoresistance. Mechanistic studies demonstrated that RBFOX3 overexpression elevates HTERT expression, promoting GC progression. Moreover, our data indicate that RBFOX3 binds to AP-2β to promote HTERT expression. Taken together, our findings highlight the RBFOX3/HTERT signaling axis as a new therapeutic target for the treatment of GC.

## Materials and Methods

### Clinical Samples

In total, 178 paired human GC tissues and adjacent non-tumor tissues were collected from the Second Affiliated Hospital of Nanchang University. The samples had been biobanked between August 2017 and December 2019, and 92 were from males and 86 were from females. Adjacent, matched non-cancer tissues were collected >5 cm away from the edge of the cancerous foci. This research was approved by the Ethics Committee of the Second Affiliated Hospital of Nanchang University.

### Cell Lines and Antibodies

Five human GC cell lines (MGC-803, MKN45, AGS, SGC-7901, and BGC-823) and normal gastric epithelial cell line (GES-1) were purchased from the American Type Culture Collection. All cells were authenticated *via* short tandem repeat profiling by the Cell Bank and cultured in RPMI-1640 medium (Corning, 10-040-CVR), supplemented with 10% fetal bovine serum (Sigma, 12103C), in a humidified incubator at 37°C, 5% CO_2_. Rabbit anti-RBFOX3 (Abcam, ab177487) was used at 1:1,000 for Western blot and 1:3,000 for immunohistochemistry (IHC). Rabbit anti-HTERT (Abcam, ab183105) was used at 1:1,000 for Western blot and 1:100 for IHC. Mouse anti-E-cadherin (Abcam, ab1416) was used at 1:50 for Western blot, rabbit anti-β-catenin (Abcam, Ab32572) was used at 1:5,000 for Western blot, and rabbit anti-IgG (Abcam, ab2410) and rabbit anti-GAPDH (Abcam, ab9485) were used at 1:2,500 for Western blot.

### Streptavidin–Agarose Pull Down Assay

HTERT promoter binding proteins were analyzed by streptavidin–agarose pull-down assays. Nuclear proteins were extracted from GC cells and 1 mg was incubated with 10 μg of biotinylated double-stranded DNA probes (Sigma-Aldrich) related to −351 to −149 of the region of HTERT promoter. After adding 100 μl streptavidin–agarose beads (Sigma-Aldrich), the cells were pulled down by centrifuging at 500 *g* at 4°C for 10 min.

### Spectrometry Assay

Using mass spectrometry assay, HTERT promoter-binding proteins were analyzed. Then, the binding proteins were separated by 10% sodium dodecyl sulfate-polyacrylamide gel electrophoresis (SDS-PAGE) and observed by silver staining (Beyotime, P0015A). After reduction and alkylation, the bands of interest were digested with MS-grade trypsin solution (Promega, CAS9002-07-7). We used mass spectrometry to identify the digested peptides. The identities of the proteins were detected by software.

### Transient Transfection

Cell transfection was conducted by the use of Lipofectamine 3000 (Invitrogen CA, USA). PcDNA3.1-RBFOX3 and pcDNA3.1-AP-2β plasmids and shRBFOX3 (5′-CAAATCGGGGGGTTGCCAA-3′ and 5′-ACCGTGACCTCGCTCAAAT-3′) and siAP-2β (5′-GCAGUCCAAUGACAUUUGATT-3′) were purchased from GenePharma (Shanghai, China).

### Chromatin Immunoprecipitation Assay

The cells were fixed with 1% formaldehyde and then cross-linking quenched with 100 μl of 1.375 M glycine/ml of cell culture media. Then, these were sonicated on ice to shear DNA into 200–900-bp fragments (setting parameters of the ultrasound machine: 30% power, turn on 2 s, interval 3 s, 4 min). A third of the cell lysate was used as DNA input control, a third was used for immunoprecipitation with anti-RBFOX3 antibodies, and a third was subjected to non-immune rabbit IgG (Cell Signaling Technology, 3900S). The DNA fragments were purified on spin columns (Qiagen, 31014) and used to amplify a 227-bp segment of the HTERT promoter region using the following primers: Fwd: 5′-TGGCCTTCCCCAGGGCCCTTC-3′, Rvs: 5′-TGAGGACG GGCAGGGAGTGC-3′.

### Lentiviral Construction and Cell Transfection

Overexpressing RBFOX3 and U6-sh-RBFOX3-EGFP-IRES-puromycin were designed and synthesized by Genechem, Shanghai, China. We then selected stable clones after 2 weeks by treating the cells with 0.7–5 μg/ml puromycin. After clonal expansion, we quantified the RBFOX3 expression by RT-qPCR and Western blotting. Cell transfection was conducted by the use of Lipofectamine 3000 (Invitrogen CA, USA). Silencing efficiency was analyzed by RT-qPCR and Western blotting.

### Colony Formation and 5-Ethynyl-20-Deoxyuridine Assays

Colony formation assays were performed as we previously described (15). The transfected GC cells were seeded in six-well plates at a density of 1 × 10^5^ cells/well. A total of 100 μl of 10 uM prewarmed Edu was added into each well and cultured for 2 h. After adding 4% paraformaldehyde for 15 min, 50 μl of 2 mg/ml glycine solution was decolorized for 5 min. The cells were permeabilized with 0.3% Trix-100 PBS for 10 min, followed by Apollo and Hoechst staining. Finally, they were examined by confocal microscopy.

### Wound Healing and Transwell Assays

The transfected GC cells were seeded in six-well plates and then imaged 0 and 24 h later to monitor migration. These experiments were performed as independent triplicates. Transwell assays were used in BD BioCoat matrigel invasion chambers (BD, 354480). The invading cells in five randomly selected fields of view were observed under the microscope.

### Western Blot

The collected cells were prepared using complete Lysis-M reagent (Roche, 4719956001) and RIPA lysis buffer (Beyotime, P0013B). Protein concentration was detected by the bicinchoninic acid assay (ThermoFisher Scientific, 23,221–23,230). The protein was separated by using 8–10% SDS-PAGE and 0.45-μm PVDF membranes, with antibody staining, and analyzed.

### Real-Time PCR

Total RNA was done using TRIZOL reagent (Invitrogen, 15596-026) as per the manufacturer's instructions. cDNA synthesis was carried out using ReverTra Ace qPCR RT kit (Toyobo, FSQ-201C). RT-qPCR was done using a SYBR Green PCR kit (Toyobo, KGA1339-1) on a Bio-Rad CFX96 machine. The results were analyzed by using the 2^−ΔΔCT^ method. These experiments were done as independent triplicates. All the primers were designed by GeneCopoeia.

### Co-immunoprecipitation Assay

The cells in each group were collected with the indicated antibodies and then added with 50 μl of agarose-conjugated protein-A/G beads (Merck Millipore, YB36403ES03) at 4°C overnight. Using PBS 1 × washing with ice, the loading buffer was added into the beads and heated at 4°C for 5 min. Finally, they were examined by Western blot.

### *In vivo* Tumor Growth Assay

The nude mice (6–8 weeks old) were purchased from Shanghai Laboratory Animal Co., Ltd. The SGC-7901 cells expressing luciferase reporter (pcDNA3.1-luciferase) were stably transfected with shRBFOX3 and pLVTHM. Next, about 1 × 10^6^ of SGC-7901 cells (mixed beforehand with Matrigel, 1:1) were carefully injected into the subrenal capsule. The IVIS system (Caliper Life Sciences) was used to detect tumor growth and metastases. After 6 weeks, the mice were sacrificed and the tumors were collected for analyses.

### Statistical Analysis

Data are presented as mean ± SD of three independent experiments. SPSS 11.0 software was used for processing of the statistical data. *P* < 0.05 was considered as statistically significant.

## Results

### RBFOX3 Is Overexpressed in GC Tissues and Positively Correlates With Tumor Progression

To identify the abnormally expressed RBFOX3 in GC tissues, *RBFOX3* DNA digestion products were first identified by agarose gel electrophoresis. The DNA digestion products were then stably expressed in GC cells (Figure 1A). The RT-qPCR assay revealed that RBFOX3 was consistently elevated in GC tissues (*p* < 0.001, Figure 1B). The IHC analyses of 89 GC tissues and non-tumor tissues showed higher RBFOX3 staining in the GC tissues relative to controls (*p* < 0.01, Figure 1C). Similar observations were obtained in a Western blot assay performed on 37 frozen GC tissues and non-tumor tissues (*p* < 0.05, Figure 1D). The Western blot analysis of cell lines revealed that RBFOX3 was down-regulated in GES-1 cells relative to the GC cells (Figure 1E). Next, we evaluated the relationship between the RBFOX3 level and the clinicopathological features of GC (Table 1). This analysis indicated that the high level of RBFOX3 was associated with tumor differentiation (*p* = 0.017), AJCC clinical stage (*p* = 0.015), and TNM stage (*p* = 0.004). A Kaplan–Meier survival analysis revealed significantly lower overall survival (OS) and disease-free survival (DFS) rates in patients with high tumor RBFOX3 levels relative to those expressing low RBFOX3 levels (Figures 1F,G). The univariate and multivariate Cox regression analyses also showed that advanced TNM stage and high RBFOX3 expression significantly correlated with unfavorable OS and DFS. Taken together, these results showed that a high level of RBFOX3 is associated with poor prognosis, indicating that RBFXO3 could be an independent prognostic marker in GC (hazard ratio = 2.670; 95% CI, 1.471–3.917; *p* = 0.001; Table 2).

**Figure 1:** High RBFOX3 protein expression predicted a dismal prognosis of gastric cancer (GC) patients. **(A)** RBFOX3 DNA digested fragment expression was examined *via* agarose gel electrophoresis in SGC-7901 as well as MGC-803 cells. **(B)** RT-qPCR was conducted in GC tissue samples (*n* = 47) and the corresponding precancerous tissue samples (*n* = 47) to determine RBFOX3 mRNA expression. **(C)** Representative images showing the immune-histochemical findings of RBFOX3 in normal gastric mucosa and GC tissues (*n* = 89). **(D)** The expression of RBFOX3 protein in 37 human GC tissues and the adjacent tissues as detected by Western blot analysis. **(E)** The protein expression level of RBFOX3 in normal gastric epithelial cells (GES-1) compared with GC cell lines (MKN45, AGS, SGC-7901, MGC-803, and BGC-823). **(F,G)** Kaplan–Meier survival analysis of the overall survival and the disease-free survival in the two groups designated by low and high expression of RBFOX3 in patients with GC.

**Table 1:** Correlation of the expression of RBFOX3 with clinical features in gastric cancer.

**Characteristics**	**RBFOX3 expression**		***p*-value**
	**Low group** **(*N =* 89)**	**High group** **(*N =* 89)**	
Age (y)			*p* = 0.759
<60	36	33	
≥ 60	53	56	
Gender			*p* = 0.294
Male	42	50	
Female	47	39	
Diameter (cm)			*p* = 0.122
<5	50	61	
≥ 5	39	28	
Location			*p* = 0.552
Proximal	24	24	
Middle	21	27	
Distal	44	38	
Differentiation			***p*** **=** 0.017^*^
Poor	23	41	
Moderately	29	19	
Highly	37	29	
Lauren type			*p* = 0.563
Intestinal	71	74	
Diffuse or mixed	18	15	
AJCC clinical stage			***p*** **=** 0.015^*^
I	49	37	
II + III	40	62	
Drinking alcohol			*p* = 0.118
No	20	12	
Yes	69	77	
Smoking			*p* = 0.563
No	18	15	
Yes	71	74	
TNM stage			***p*** **=** 0.004^**^
I + II	50	31	
III + IV	39	58	
Lymphatic metastasis			*p* = 0.602
N0 + N1	44	38	
N2	25	26	
N3	20	25	

* p < 0.05,

** *p < 0.01*.

**Table 2:** Univariate and multivariate regression analyses of parameters associated with prognosis of GC patients.

**Characteristics**	**Subset**	**Univariate analysis**		**Multivariate analysis**	
		***p*-value**	**HR (95% CI)**	***p*-value**	**HR (95% CI)**
Age	<60/≥ 60	0.137	1.354 (0.968–1.994)	–	–
Gender	Male/female	0.741	0.931 (0.338–1.835)	–	–
Diameter	<5 cm/≥ 5 cm	0.630	1.335 (0.634–2.567)	–	–
Location	Proximal/Middle/Distal	0.224	1.016 (0.512–2.016)	–	–
Drinking alcohol	No/Yes	0.318	2.445 (1.145–5.345)	–	–
Smoking	No/Yes	0.377	8.474 (1.223–52.031)	–	–
Lauren	Intestinal/Diffuse or mixed	0.914	0.527 (0.361–1.158)	–	–
Lymphatic metastasis	N0 + N1/N2 + N3	0.506	0.716 (0.434–1.098)	–	–
Differentiation	Poor + Moderately/Highly	0.014^*^	1.204 (0.432–1.943)	0.062	1.341 (1.015–2.578)
Ajcc clinical stage	I + II/III	0.001^**^	2.179 (1.588–3.493)	0.129	4.083 (0.549–10.240)
TNM stage	I + II/III + IV	0.002^**^	3.118 (2.090–5.567)	0.006^**^	2.118 (0.837–4.651)
RBFOX3	High/Low	0.001^**^	3.521 (2.084–4.747)	0.001^**^	2.670 (1.471-3.917)

* p < 0.05,

** *p < 0.01*.

### RBFOX3 Promotes GC Cell Proliferation and Cell Cycle Progression *in vitro*

To explore the function of RBFOX3 in GC cell growth, RBFOX3 was stably overexpressed in SGC-7901 cells and stably silenced in MGC-803 cells. The results showed that the up-regulation of RBFOX3 markedly increased SGC-7901 cell viability and colony formation (*p* < 0.05, Figures 2A,D). RBFOX3 silencing effectively suppressed the MGC-803 cell viability and colony formation (*p* < 0.05, Figures 2B,E). Interestingly, the effect of RBFOX3 knockdown was reversed by HTERT overexpression in MGC-803 cells (*p* < 0.05, Figures 2C,F). Flow cytometry revealed that RBFOX3 silencing remarkably arrested MGC-803 cell cycle at the G1 phase (*p* < 0.05, Figure 2H). RBFOX3 overexpression in SGC-7901 cells had similar results (*p* < 0.05, Figure 2G). Taken together, these results indicate that RBFOX3 increases the proliferation of GC cell *in vitro*.

**Figure 2:** RBFOX3 promoted gastric cancer (GC) cell multiplication and cell cycle progression *in vitro*. **(A,D)** RBFOX3 overexpression increased the propagative viability of cells as well as the formation of colonies in SGC-7901 cells. **(B,E)** RBFOX3 silencing decreased the viability of cells as well as the capacity of formation of colonies in MGC-803 cells. **(C,F)** Overexpression of HTERT reverted the repression of viability of cells and colony formation moderated by the silencing of RBFOX3 in MGC-803 cells. **(G,H)** Flow cytometric analyses of the cell cycle of the indicated GC cells transfected with Vector/RBFOX3 and sh-NC/shRB-1/shRB-2. *p < 0.05, **p < 0.01.

### RBFOX3 Regulates GC Cell Migration and Invasion *in vitro*

Previous studies have reported that the HTERT signaling pathway plays an important role in cell migration and invasion (16–18). Therefore, we used wound healing and transwell invasion assays to explore the role of RBFOX3 on GC cell migration and invasion. The results showed that up-regulated RBFOX3 enhanced SGC-7901 cell migration and invasion. Conversely, RBFOX3 silencing suppressed MGC-803 cell migration (*p* < 0.05, Figures 3A,B,D,E). Moreover, HTERT overexpression in RBFOX3-silenced MGC-803 cells leads to higher migration and invasion abilities (*p* < 0.05, Figures 3C,F). To elucidate the factors driving RBFOX3-mediated metastasis, we evaluated the expression of some oncogenes and tumor suppressors in RBFOX3 knockdown (sh-RB and MGC-803) and overexpression (RBFOX3 and SGC-7901) contexts. Moreover, E-cadherin, an important protein involved in tumor metastasis, was downregulated, while β-catenin was markedly elevated upon RBFOX3 overexpression (SGC-7901 cells) (*p* < 0.05, Figure 3G), suggesting that perturbation in the expression of these proteins may be associated with RBFOX3 and mediate GC processes. An opposite effect was also observed upon RBFOX3 silencing (sh-RB and MGC-803) (*p* < 0.05, Figure 3H).

**Figure 3:** RBFOX3 promoted the migration and the invasion of GC cells *in vitro*. **(A–C)** The wound healing assay was performed to investigate the horizontal migration of cells following RBFOX3 overexpression or silencing in SGC-7901 (left panel) and MGC-803 cells (middle panel). Overexpression of HTERT abolished the inhibitory effects of RBFOX3 silencing on cell viability and formation of colonies in MGC-803 cells (right panel). **(D–F)** Results of the vertical migration and the invasion capacities of cells following RBFOX3 overexpression or silencing in SGC-7901 (left panel) and MGC-803 (middle panel) cells. **(G,H)** Western blotting results showing the protein expression of metastasis-related proteins following RBFOX3 overexpression or silencing in SGC-7901 and MGC-803 cells. *p < 0.05, **p < 0.01, ***p < 0.001.

### RBFOX3 Inhibition Enhances 5-Fu Sensitivity in GC Cells

Although 5-fluorouracil (5-Fu) is commonly used to treat GC, it is associated with negative side effects (19). We hypothesized that, given the effect of RBFOX3 on GC growth and proliferation, its knockdown might enhance GC sensitivity to 5-Fu. We observed that 5-Fu inhibited GC cell viability and colony formation in a dose-dependent manner. Additionally, these effects were significantly stronger in the background of RBFOX3 silencing (*p* < 0.05, Figure 4A). Next, we first generated MGC-803 stably expressing RBFOX3 shRNA (shRB-1 and shRB-2) or the negative control (sh-NC). We found that the cell viability of RBFOX3 knockdown cells treated with 5-Fu was significantly lower relative to that of mock knockdown cells treated with 5-Fu (*p* < 0.05, Figure 4B). Moreover, RBFOX3 expression decreased after adding 5-Fu (*p* < 0.05, Figure 4C). This suggested that RBFOX3 regulated GC cell sensitivity to 5-Fu. However, their specific mechanism needs further research to fully reveal how RBFOX3 regulates sensitivity to 5-Fu.

**Figure 4:** RBFOX3 regulated the sensitivity of GC to 5-Fu. **(A)** A representative image showing the results of clonogenic assay in MGC-803 cells following RBFOX3 knockdown or control groups. The graph denotes the mean of number of colonies ± SD with respect to the vehicle control, three biological replicates with two technical replicates; two-way analysis of variance with Dunnett's multiple-comparison test. DMSO, dimethyl sulfoxide. **(B)** The effect of RBFOX3 repression on the response of MGC-803 cells to 5-Fu treatment. Data are shown as means ± SEM for three biological replicate experiments with three technical replicates. We transfected the MGC-803 cells with RBFOX3 shRNA (shRB-1 and shRB-2). We measured the viability of cells using the MTS assay with or without 5-Fu treatment with respect to time. **(C)** Western blot results showing the expression of RBFOX3 protein in MGC-803 cells treated with DMSO/10 nM/30 nM 5-Fu arms and in control cells. *p < 0.05, **p < 0.01.

### RBFOX3 Binds to the HTERT Promoter in GC Cells

Previous studies have identified regulatory factors associated with the HTERT promoter in lung and liver tumors using streptavidin–agarose bead pull-down assays (17, 20). To establish whether RBFOX3 interacts with the HTERT promoter in GC as well, we used 5′-biotinylated HTERT promoter probes and streptavidin–agarose beads in GC cells to pull down cytoplasmic proteins bound to the HTERT promoter. We then used RBFOX3 antibody to detect the location of RBFOX3 in the cytoplasmic protein/DNA complex by Western blot. RBFOX3 bound to the HTERT promoter probe in GC cells (MKN45, AGS, SGC-7901, MGC-803, and BGC-823) (Figure 5A, upper panel). All the GC cell lines express high levels of RBFOX3 (Figure 5A, lower panel). We used chromatin immunoprecipitation (ChIP) assay to analyze the relationship between RBFOX3 and HTERT. The results showed that RBFOX3 bound to the HTERT promoter in GC cells (Figure 5B). We designed three different 5′-biotinylated HTERT promoter fragments to explore the binding site of RBFOX3 on the HTERT promoter (Figure 5C). The results of this test indicated that the −371 to −305 (5′-C GCTGACCCCACCGTTCTAGGCAAGGCGTTCACCCGCCCTCTTGGGGCCCTCGCTGGCGTCCCTGC-3′) region of the HTERT promoter is critical to the binding of RBFOX3. To investigate whether RBFOX3 regulates HTERT expression, we constructed plasmids with overexpressed RBFOX3, and shRBFOX3. The Western blot result revealed that up-regulated RBFOX3 increased HTERT expression, while down-regulated RBFOX3 inhibited HTERT expression in GC cells (*p* < 0.05, Figures 5D,E). HTERT siRNA silencing did not significantly affect RBFOX3 expression (Figures 5F,G). Next, we investigated how elevated RBFOX3 and HTERT expression in GC tissues (*n* = 52) affects the clinical outcomes. We observed that RBFOX3 expression was positively correlated with HTERT in GC tissues (Figures 5H,I). These results were consistent with those shown in Figures 5D–G. To investigate the relationship between RBFOX3 and HTERT, we restored RBFOX3 expression in lentivirus-stabilized RBFOX3 knockdown in SGC-7901 cells. The results showed that RBFOX3 overexpression restored RBFOX3 and HTERT expression (*p* < 0.05, Figure 6A). Similar results were obtained in MGC-803 cells with stably silenced RBFOX3 expression (*p* < 0.05, Figure 6B). Additionally, RBFOX3 overexpression restored cell proliferation, viability, and invasion capacity (*p* < 0.05, Figures 6C–**H**). These findings altogether confirm that RBFOX3 regulates HTERT expression.

**Figure 5:** RBFOX3 functioned as a HTERT promoter binding protein in gastric cancer (GC) cells. **(A)** We detected the binding of RBFOX3 on the 5′-biotin-labeled HT ERT promoter probe or a non-specific probe (NSP) *via* Western blot using anti-RBFOX3 antibody. We detected RBFOX3 protein in the cytoplasm protein-HTERT probe-streptavidin bead complexes in MKN45, AGS, SGC-7901, MGC-803, and MGC-823 cells (upper panel). We analyzed the expression of total RBFOX3 proteins in GC cells using Western blot and utilized tubulin as a loading control (lower panel). **(B)** Chromatin immunoprecipitation assays were conducted in GC cells using RBFOX3 antibody and HTERT promoter primers. We separated the PCR products on 2% agarose gels. We used IgG as a negative control. **(C)** We incubated the 5′-biotin-labeled probes corresponding to the diverse fragments of HTERT promoter (probes 1–3, left panel) or a non-specific probe with MGC-803 cell lysates and streptavidin beads. Western blot results using anti-RBFOX3 antibody (right panel) show the detection of the protein-bound proteins. **(D,E)** HTERT protein expression was down-regulated in RBFOX3-silenced SGC-7901 as well as MGC-803 cells and up-regulated in RBFOX3 overexpressing SGC-7901 and MGC-803 cells. **(F,G)** RBFOX3 protein expression was not affect in HTERT-silenced SGC-7901 as well as MGC-803 cells. **(H)** Immuno-histochemical results of RBFOX3 and HTERT protein levels from GC tissues represented by two images. “Low” denotes the low expression of both RBFOX3 and HTERT and “High” denotes the high protein expression of both RBFOX3 and HTERT. **(I)** Association between the expressions of RBFOX3 and HTERT in 37 GC paraffin section samples from GC tissues. Pearson correlation test, *n* = 37, *r* = 0.419, *p* = 0.005. *p < 0.05, **p < 0.01.

**Figure 6:** RBFOX3 promotes gastric cancer multiplication and invasion by up-regulating HTERT expression. **(A)** The silencing of HTERT (siHTERT-1) repressed the up-regulation of HTERT expression in SGC-7901-RBFOX3 cells. **(B)** Overexpression of HTERT (pcDNA3.1-HTERT) attenuated the HTERT expression in MGC-803-shRB cells. **(C–H)** Colony formation, Edu, and invasion assays showing that the knockdown or the overexpression of ectopic HTERT significantly rescues the RBFOX3-overexpressed or RBFOX3-silenced cell division and invasion observed in SGC-7901 and MGC-803 cells. *p < 0.05, **p < 0.01.

### RBFOX3 Interacts With AP-2β to Regulate HTERT Expression

This study investigated whether RBFOX3 bound to the HTERT promoter interacted with other transcription factors. Previous studies showed that the HTERT promoter-binding proteins include KLF4 (21), RFPL3 (22), CPSF4 (23), and AP-2β (17). To test this possibility, we performed a Co-IP pull-down experiment and, using a RBFOX3-specific antibody, observed that RBFOX3 bound to AP-2β (Figures 7A,B). Interestingly, we found that AP-2β bound to the HTERT promoter (Figure 7C). A co-immunofluorescence analysis of GC cells revealed that RBFOX3 and AP-2β were primarily localized in the nucleus and co-localized (Figure 7D). Additionally, we found that AP-2β increased the ability of RBFOX3 binding to the HTERT promoter (Figures 7E,G). Conversely, AP-2β knockdown weakened this binding even in the context of RBFOX3 overexpression (SGC-7901 cells) (Figures 7E,G). A luciferase reporter analysis showed that the up-regulation of AP-2β enhanced the activity of the HTERT promoter, while the down-regulation of AP-2β inhibited the activity of the HTERT promoter (Figure 7G). To investigate the influence of AP-2β on HTERT, we performed Western blot analysis and found that AP-2β overexpression enhanced HTERT expression. Conversely, AP-2β knockdown suppressed HTERT expression (Figure 7F) as well as abolished the inhibition of AP-2β knockdown on the invasion of GC cells. Conversely, AP-2β overexpression partially rescued the inhibition of GC invasion caused by the RBFOX3 knockdown (Figure 7H). These findings suggest that RBFOX3 bound to AP-2β and then regulated the HTERT expression in GC cells.

**Figure 7:** RBFOX3 interacted with AP-2β and modulated the expression of HTERT. **(A,B)** We transfected SGC-7901 cells with RBFOX3 overexpression or empty vector. CoIP analysis was used to detect the interaction between RBFOX3 and AP-2β. **(C)** We performed the chromatin immunoprecipitation (ChIP) assays using the antibody against AP-2β. We separated the PCR products of the HTERT promoter (−378 to −157) on 2% agarose gels. **(D)** We cultured the SGC-7901 as well as the MGC-803 cells grown on chamber slides for 24 h and examined the subcellular localization and the co-localization of RBFOX3 with AP-2β *via* confocal microscopy analysis. **(E)** We performed the ChIP assays using the HTERT promoter primers and the respective RBFOX3 antibodies in SGC-7901 cells transfected with RBFOX3, RBFOX3, and siAP-2β, AP-2β, AP-2β, and shRBFOX3, respectively. **(F)** The expression of HTERT in SGC-7901 cells transfected with RBFOX3, RBFOX3, and siAP-2β, AP-2β, AP-2β, and shRBFOX3, respectively. **(G)** Relative HTERT promoter activity in SGC-7901 cells transfected with RBFOX3, RBFOX3, and siAP-2β, AP-2β, AP-2β, and shRBFOX3, respectively. **(H)** We performed the Transwell invasion assay in SGC-7901 cells transfected with RBFOX3, RBFOX3, and siAP-2β, AP-2β, AP-2β, and shRBFOX3, respectively. *p < 0.05, **p < 0.01.

### Deregulation of RBFOX3 Suppresses Tumor Growth in GC Orthotopic Xenografts

To evaluate whether RBFOX3 has oncogenic functions, we established GC orthotopic mouse xenografts using SGC-7901 cells carrying a luciferase reporter and stably overexpressing RBFOX3, as well as MGC-803 cells carrying the luciferase reporter and stable knock-down of RBFOX3. As controls, we used vector groups and sh-NC groups, respectively. The cells were inoculated in the renal capsule of the mouse (eight mice per group). Tumor growth was monitored using IVIS. At 6 weeks into the experiment, we observed that RBFOX3 knockdown resulted in significantly smaller tumors, while RBFOX3 overexpression resulted in tumors that were significantly bigger than the controls (Figures 8A,D). An analysis of tumor size revealed that RBFOX3 up-regulation significantly promoted tumor volume and weight (Figures 8B,C). However, the knock-down of RBFOX3 produced opposite effects (Figures 8E,F). These findings show that the down-regulation of RBFOX3 may suppress tumor progression *in vivo*.

**Figure 8:** Dysregulation of RBFOX3-suppressed cell multiplication in gastric cancer (GC) orthotopic xenografts. Stable transfection of the SGC-7901 and MGC-803 cells with pcDNA3.1-RBFOX3 plasmid or empty plasmid (Vector) and RBFOX3 shRNA or negative control vector (sh-NC), respectively. Next, we subcutaneously injected the transfected GC cells into nude mice, and xenograft tumor growth was determined for 25 days. **(A–C)** IVIS representative images showing the tumor size **(A)**, growth curves of tumor volumes **(B)**, and tumor weight **(C)** in RBFOX3 overexpressed arm *vs*. control arm. **(D–F)** IVIS representative images showing the tumor size **(D)**, growth curves of tumor volumes **(E)**, and tumor weight **(F)** in shRB-1 arm *vs*. controls. *n* = 8, *p < 0.05, **p < 0.01.

## Discussion

Limitless self-renewal is a hallmark of cancer (24). Telomere maintenance and telomerase activation have been reported to promote the proliferation of cancer cell (25). The transcriptional regulation of HTERT is believed to modulate telomerase activation in human cancers. Particularly, HTERT maintains telomere length, thereby overcoming senescence and hence modulating cancer development (26, 27). HTERT is up-regulated in various tumors, and it influences tumor development *via* genetic and epigenetic mechanisms such as HTERT promoter mutations, HTERT amplifications, HTERT promoter methylation, and HTERT structural variation (28, 29). HTERT is the catalytic subunit of telomerase which plays crucial roles in the cells' unlimited replication (29–31). Recent findings have implicated HTERT in various human diseases, including cancer (17, 30, 32). Recently, HTERT is often maladjusted, which is considered as a cancer hallmark and a potential therapeutic target (30, 31, 33). The differentially expressed tumor-specific cytokines bind to the HTERT promoter to promote HTERT expression and the development of cancer (32, 34). Interestingly, we found that RBFOX3 is markedly up-regulated in GC tissues and cell lines and functions as an oncogene. Our data showed that patients expressing high RBFOX3 levels exhibit significantly shorter OS and DFS. Furthermore, the univariate and multivariate analyses showed that a high RBFOX3 expression may independently predict poor GC prognosis.

Next, we investigated the significance of high RBFOX3 expression in GC. A functional analysis revealed that RBFOX3 overexpression promoted GC cell proliferation and metastasis. However, the effects of RBFOX3 overexpression on GC cells are suppressed by RBFOX3 silencing. We also established that RBFOX3 influenced GC cell sensitivity to 5-Fu. It has been reported that RBFOX3 can bind to the region of the HTERT promoter, thereby regulating HTERT signaling (17, 33). Interestingly, we find that the inhibitory effects of RBFOX3 knockdown in GC proliferation and invasion were rescued by HTERT overexpression.

Next, we investigate whether RBFOX3 also bound to the region of the HTERT promoter in GC cells. We performed biotin–streptavidin–agarose pull-down and proteomics analysis, which revealed that RBFOX3 functioned as a novel HTERT promoter-binding protein in GC cells. Importantly, we found that RBFOX3 could bind to the region of the HTERT promoter in GC cells and activate it. Additionally, our data showed that RBFOX3 could regulate the HTERT expression at the transcriptional level. Further analysis demonstrated that RBFOX3 was up-regulated in primary human GC cells. To further investigate the mechanism of RBFOX3 regulation of HTERT, we constructed RBFOX3 stably overexpressing plasmids and RBFOX3 stable knockdown in GC cells using a lentivirus carrying shRNA. A Western blot analysis revealed that RBFOX3 overexpression elevated the HTERT protein levels in GC cells, while its silencing inhibited HTERT expression at the translational level in GC cells. Furthermore, we explored the impact of elevated RBFOX3 on HTERT in GC clinical outcomes. The results showed that RBFOX3 correlated with HTERT expression in GC tissues relative to matching paracancerous tissues. RBFOX3 and HTERT were correlated with advanced disease and could be a poor prognosis in GC patients.

To further verify the effects of RBFOX3 in HTERT, we restored RBFOX3 expression in stably silenced GC cell lines. This restored RBFOX3 and HTERT expression in SGC-7901 and MGC-803 cells. However, HTERT silencing did not alter the RBFOX3 levels; it restored cell proliferation and invasion. These results revealed that RBFOX3 regulated the HTERT expression.

Finally, we observed that RBFOX3 binds to AP-2β to promote the expression of HTERT and confirmed, through ChIP assay, that AP-2β bound to the HTERT promoter. AP-2β overexpression enhanced RBFOX3 binding to the HTERT promoter. Conversely, the down-regulation of AP-2β inhibited RBFOX3 binding to the HTERT promoter, with the RBFOX3 overexpressing in SGC-7901 cells. The luciferase reporter assay revealed that AP-2β overexpression increased the activity of the HTERT promoter, an effect that was inhibited following AP-2β knockdown. In further tests, we found that AP-2β up-regulated HTERT, while AP-2β knockdown down-regulated the HTERT expression. The MTS assay analysis revealed that the knockdown of AP-2β inhibited the RBFOX3 overexpression-mediated GC cell growth. Moreover, AP-2β overexpression partially rescued the inhibitory effects of RBFOX3 knockdown growth. These data altogether showed that RBFOX3 regulated HTERT expression and GC cell growth through binding to AP-2β.

Although RBFOX3 is an antigen of the neuronal marker antibody NeuN (35), it has been implicated in GC. Recent studies indicate that RBFOX3 regulates various physiological processes apart from being an alternative splicing factor (17, 36). It binds DNA and regulates microRNA transcription (12, 14). However, its role in mammalian development and homeostasis has remained unclear. RBFOX3 possesses an RNA recognition motif-type RNA binding domain which enables it to regulate splicing events by binding the (U)GCAUG sequence on RNA (14, 37). Here we find that RBFOX3 can regulate the expression of HTERT through binding to the HTERT promoter in GC cells. However, the role of RBFOX3 in the processes of RNA binding is not clear.

In summary, we reveal that RBFOX3 can function as an oncogene to promote GC cell proliferation, migration, and invasion. Furthermore, we have shown that RBFOX3 also activates HTERT signaling through AP-2β in GC cells. Thus, our study provides a novel thought in the regulation of HTERT in the progress of GC, and RBFOX3 is a novel therapeutic target against GC.

## Data Availability Statement

The raw data supporting the conclusions of this article will be made available by the authors, without undue reservation, to any qualified researcher.

## Ethics Statement

The studies involving human participants were reviewed and approved by Medical Research Ethics Committee of the Second Affiliated Hospital of Nanchang University. The patients/participants provided their written informed consent to participate in this study. The animal study was reviewed and approved by Medical Research Ethics Committee of the Second Affiliated Hospital of Nanchang University. Written informed consent was obtained from the owners for the participation of their animals in this study. Written informed consent was obtained from the individual(s) for the publication of any potentially identifiable images or data included in this article.

## Author Contributions

ZZh, CL, and XZ: project design and conception. CL, XZ, QL, FB, CHua, KL, JZhu, WZ, ZZo, HL, JH, CHu, and JZha: performed the research and data collection. XZ, CL, and FB: data statistical and analysis. XZ and CL: drafted the manuscript. All authors read and approved the final version of the manuscript.

## Conflict of Interest

The authors declare that the research was conducted in the absence of any commercial or financial relationships that could be construed as a potential conflict of interest.
